# Colonic flora, Probiotics, Obesity and Diabetes

**DOI:** 10.3389/fendo.2012.00087

**Published:** 2012-07-11

**Authors:** Paul E. Marik

**Affiliations:** Division of Pulmonary and Critical Care Medicine, Department of Medicine, Eastern Virginia Medical School,Norfolk, VA, USA

**Keywords:** probiotics, obesity and diabetes

## Abstract

Obesity results from alterations in the body’s regulation of energy intake, expenditure, and storage. Animal and human data demonstrate that phylogenic changes occur in the microbiota composition in obese individuals. Furthermore, evidence from animal models suggest that the alterations of the gut microbiota with obesity results in increased energy extraction and lipid deposition, altered release of entero-hormones, increased intestinal permeability and metabolic endotoxemia. Treatment with pre- and probiotics may reverse many of metabolic effects linked with the altered microbiota in obese patients. The gut microbiota is, therefore, a potential nutritional and pharmacological target for the management of obesity and obesity-related disorders.

Mammals, including humans, have, throughout their evolution, been associated with complex microbial communities, which inhabit the surfaces and alimentary tract of their host and which outnumber the human somatic cells by a factor of 10. The human intestinal microbiota is estimated to be composed of 10^13^ to 10^14^ microorganisms whose collective genome, the microbiome, contains at least 100-fold more genes than the complete human genome (Eckburg et al., 2005; Gill et al., 2006). The gut of a neonate is sterile. However, at birth, the gut is immediately colonized by maternal and environmental bacteria and the complexity of the resulting gut microbiota increases until weaning to solid foods. Although incompletely understood the gut microbiota is implicated in a variety of host functions involving intestinal development and function, including epithelial turnover, immune modulation, gastrointestinal motility, and drug metabolism. The gut microbiota also has important metabolic functions, breaking down dietary toxins and carcinogens, synthesizing micronutrients, fermenting indigestible food substances, assisting in the absorption of certain electrolytes and trace minerals, and affecting the growth and differentiation of enterocytes and colonocytes through the production of short-chain fatty acids (SCFA; Macfarlane and Macfarlane, 1997; Zoetendal et al., 2001; Ouwehand et al., 2002; Stappenbeck et al., 2002). Finally, the normal gut microbiota helps prevent luminal colonization by pathogenic bacteria, such as *Escherichia coli*, *Clostridia*, *Salmonella*, and *Shigella* species.

The composition of the adult intestinal microbiota has been intensively studied, by means of culture-based methodologies and,more recently, through culture independent technologies based on the amplification and direct sequencing of small subunit ribosomal DNA sequences. Among the novel investigative methods that are used to study the microbial ecology of complex bacterial communities, the so-called metagenomics approach is considered to represent the method that produces results of “gold standard” quality (Eckburg et al., 2005; Gill et al., 2006). Metagenomics is the study of microbial communities through sequence-based, compositional and/or functional analyses of all the combined microbial genomes contained within an environmental sample. With respect to its application to human intestinal microbiota, metagenomic studies of mucosal as well as fecal samples revealed the presence of representatives of the phylogenetic groups Firmicutes, Bacteroidetes, Proteobacteria, Fusobacteria, Verrucomicrobia, and Actinobacteria (Eckburg et al., 2005; Gill et al., 2006; See** Table 1)**. With a relative abundance of 25 and 65%, respectively, the two dominant phyla *Bacteroidetes* and *Firmicutes* represent together up to 90% of the total microbiota, whereas *Actinobacteria*, *Proteobacteria*, and *Fusobacteria* are the subdominant phyla with a relative abundance of about 5, 8, and 1%, respectively (Candela et al., 2010). At least 1800 genera and 16,000 phylotypes at the species level have been so far identified, and an even greater diversity at the species level has been predicted. The bacterial phyla are unevenly distributed along the length of the gastrointestinal tract. Metagenomic analyses of jejunum samples reveal a distinctive community composition which includes an abundance of bacteria belonging to the *Streptococcus* genus, whereas *Bacteroidetes* and *Firmicutes* genera are the predominant microbial groups identified in the distal ileum, ascending colon and rectum.

**Table 1:** Major Bacteria and Archaea phyla and genera found in the human gut microbiota. Reproduced with permission from DiBaise et al. (2008).

Phyla	Representative genera
**Bacteria**	
Firmicutes	*Ruminococcus*
	*Clostridium*
	*Peptostreptococcus*
	*Lactobacillus*
	*Enterococcus*
Bacteroidetes	*Bacteroides*
Proteobacteria	*Desulfovibrio*
	*Escherichia*
	*Helicobacter*
Verrucomicrobia	
Actinobacteria	*Bifidobacterium*
Cyanobacteria	*Synergistes*
**Archaea**	
Euryarchaeota	*Methanobrevibacter*

The composition of flora differs between individuals, with each person having unique strains that generally remain constant over time. Genetics, diet, immune status, infections, gastrointestinal disorders as well as antibiotics and other drugs interact to determine an individual’s unique microbiome. The effect of genotype on the composition of the human microbiota was demonstrated in a study involving monozygotic twins (Zoetendal et al., 2001). According to this report, there were greater similarities between the gut microbiota of monozygotic twins than between monozygotic twins and their unrelated marital partners. The importance of the initial colonizing microbial community on the eventual microbial composition of the gut is evident from animal studies. The composition of the mouse gut microbiota is significantly affected by maternal transmission (Ley et al., 2005). Diet is also a pivotal variable in influencing the composition of the intestinal microbiota. Studies on chemically well-defined diet components have proven a clear correlation between diet and the presence of specific bacterial groups. It has been shown that a diet rich in inulin and related fibers promote an increase in bifidobacteria, whereas the intake of dietary sulfate favors several genera of sulfate-reducing bacteria over methanogenic Archaea. Diet affects not only the microbiota composition, but more significantly the metabolic activities of the microorganisms.

Obesity results from alterations in energy balance, that is, how the body regulates energy intake, expenditure, and storage. Because starvation poses a greater danger to an organism than overabundance, our biological systems are geared to better protect against weight loss than weight gain (i.e., a *thrifty genotype*). Considerable effort has been made to improve the availability and stability of the food supply, resulting in an abundance of inexpensive, palatable, and energy-dense foods. Consequently, humans adapted for a situation of insufficiency are now confronted with the easy availability of such foods. Recent evidence suggests that the gut microbiota affect nutrient acquisition and energy regulation and that obese and lean people have differences in their gut microbial landscape. These findings raise the possibility that the gut microbiota may have a role in the development of obesity (See** Figure 1**; DiBaise et al., 2008; Cani and Delzenne, 2009).

**FIGURE 1:** ** Proposed mechanism whereby alteration of the bowel flora with a high-fat low-fiber diet alters the microbiota leading to metabolic endotoxemia with increased lipid storage and decreased insulin sensitivity.** Adapted with permission from Cani and Delzenne (2009).

In an elegant series of experiments, Backhed et al. (2004) found that young conventionally reared mice have a 40% higher body fat content than germ-free mice (gnotobiotic mice) even though they consumed less food than their germ-free counterparts. The distal gut microbiota from the normal mice were then transplanted into the gnotobiotic mice (a process known as conventionalization), resulting in a 60% increase in body fat within 2 weeks without any increase in food consumption or obvious differences in energy expenditure. The authors proposed that the gut microbiota promotes intestinal monosaccharides absorption, energy extraction from non-digestible food components via SCFA production through fermentation, *de novo* hepatic lipogenesis and adipocyte fatty acid storage. The gut microbiota influence the expression of host genes expressed in the intestine that control fatty acid absorption, oxidation, and storage. One such target is angiopoietin-related protein 4 (ANGPTL4), a potent lipoprotein lipase inhibitor. ANGPTL4 inhibits the uptake of fatty acids from circulating triglyceride-rich lipoproteins in white adipose and muscle tissues. Backhed et al. (2004) demonstrated that colonizing germ-free mice with gut microbiota leads to a drop in the intestinal expression of ANGPTL4. Several other proteins/systems (such as the endocannabinoid system and the tight junction protein zona occludin-1) are influenced by gut colonization and are changed upon dietary modulation of gut microbiota composition, which are implicated in the control of inflammation, gut barrier function, gut motility, nutrient oxidation, and storage (Delzenne and Cani, 2011).

Recent data suggests that SCFAs act not only as an energy substrate for the host, but also as a signaling molecule. SCFAs act as ligands for at least two G-protein-coupled receptors, GPR41 and GPR43 (Le Poul et al., 2003). Samuel et al. (2008) have demonstrated that GPR41^-^^/^^-^ mice colonized with a model of fermentative microbial community did not gain fat mass at the same extent as the wild-type littermates. On the basis that obesity and insulin resistance is associated with low-grade chronic systemic inflammation, Cani et al. (2007a) postulated another mechanism linking the intestinal microbiota to the development of obesity. They hypothesized that bacterial lipopolysaccharide (LPS) derived from Gram-negative bacteria residing in the gut microbiota acts as a triggering factor linking inflammation to a high-fat diet-induced metabolic syndrome. In a series of experiments in mice fed a high-fat diet they showed that a high-fat diet increases endotoxemia, favors an increase in the Gram-negative to Gram-positive colonizing bacteria and that chronic endotoxemia induces obesity, insulin resistance, and diabetes (See** Figure 1**; Cani et al., 2007a,b, 2009b). These authors demonstrated that modulation of the intestinal microbiota by using prebiotics in obese mice acts favorably on the intestinal barrier, lowering the high-fat diet-induced LPS endotoxemia and systemic and liver inflammation. Modulation of the gut flora with prebiotics has been demonstrated to increase glucagon-like peptide-2 (GLP-2) production in the colon. Increased GLP-2 production is associated with higher expression of ZO-1 which improves mucosal barrier function leading to a decrease of plasma LPS.

To assess the relative abundance of various types of gut bacteria in obese and lean mice, Ley et al. (2005) analyzed bacterial 16S rRNA gene sequences from the cecal microbiota of genetically obese (*ob*/*ob*) mice, their lean *ob*/+ and +/+ siblings, and their *ob*/+ mothers, all fed the same polysaccharide-rich diet. They found that the *ob*/*ob* mice had 50% fewer *Bacteroidetes* and correspondingly more *Firmicutes* than their lean littermates, a finding unrelated to differences in food consumption. Cani et al. (2007a,b) demonstrated that induced obesity in rodents markedly reduced the number of *Bifidobacterium* as well as* Bacteroides*-related bacteria. Ley et al. (2006) compared the distal gut microbiota of obese and lean human subjects and found that obese people had fewer *Bacteroides* and more *Firmicutes* than did lean control subjects. Interestingly, the authors observed that after weight loss (following a fat restricted or a carbohydrate restricted low-calorie diet), the ratio of Bacteroidetes to Firmicutes approached a lean type profile after 52 weeks of diet-induced weight loss (Ley et al., 2006). Collado et al. (2008) observed significant differences in gut microbiota composition according to the body weight during pregnancy. Interestingly, they found significantly higher numbers of *Bacteroides* group and of *S. aureus* in the overweight state compared with normal-weight women, and they established a positive correlation between the number of *Bacteroides* on the one hand, and the weight and BMI (before and over pregnancy), on the other hand. The *Bifidobacterium* group was present in higher numbers in normal weight than in overweight women and also in women with lower weight gain over pregnancy. In addition, these researchers demonstrated that overweight mothers give birth to neonates that have a decreased number of *Bifidobacteria* (Collado et al., 2010). The infants’ fecal microbial composition was related to the weight and weight gain of their mothers during pregnancy. This finding may be related to the effect of colonization at birth and/or inheritable obesogenic microbiota.

A recent paper has shown for the first time in humans that differences in the gut microbiota may precede overweight development. Kalliomaki et al. (2008) have shown that *Bifidobacterium* spp. number was higher in children who exhibited a normal weight at 7 years than in children becoming overweight. They observed that the *Staphylococcus aureus* was lower in children who maintain a normal weight than in children becoming overweight several years later. The authors proposed that *S. aureus* may act as a trigger of low-grade inflammation contributing to the development of obesity.

Gastric-bypass surgery has been shown to be very effective in reversing insulin resistance (Mingrone et al., 2012; Schauer et al., 2012). This effect has been observed to occur early after surgery and before the patients have had a significant loss of weight. It has been postulated that the surgically altered anatomy and flow of nutrients results in alteration of the microbiome which may explain this finding (Cani and Delzenne, 2011). Li et al. (2011) performed bacterial profiling to determine the effect of Roux-en-Y gastric bypass in a non-obese rat model. At 2 weeks post-surgery they noted substantial shifts of the main gut phyla toward higher concentrations of Proteobacteria (52-fold). Lower concentrations of Firmicutes (4.5-fold) and Bacteroidetes (twofold) in comparison with sham-operated rats were also found.

## EFFECT OF PREBIOTICS, PROBIOTICS, AND SYNBIOTICS ON WEIGHT LOSS AND INSULIN RESISTANCE

The best non-surgical strategy for reversing obesity in the population may be to promote small but long-term changes in diet and physical activity that take advantage of our biological systems for regulating energy balance and preventing positive energy balance. Although clearly no substitute for proper diet and exercise, manipulation of the gut microbiota may represent a novel approach for treating obesity, one that has few adverse effects.

A probiotic is defined as “*a preparation of or a product containing viable, defined microorganisms in sufficient numbers, which alter the microflora of the host and by that exert beneficial health effects in this host*” (Schrezenmeir and de Vrese, 2001). The term *prebiotic* was introduced by Gibson and Roberfroid (1995), who defined prebiotics as “*a non-digestible food ingredient that beneficially affects the host by selectively stimulating the growth and/or activity of one or a limited number of bacteria in the colon*.” The term *synbiotic* is used when a product contains both probiotics and prebiotics.

### PREBIOTICS

Prebiotic agents are non-digestible oligosaccharides that act as “fertilizers” of the colonic microbiota, enhancing the growth of beneficial commensal organisms (e.g., *Bifidobacterium* and *Lactobacillus* species; Schrezenmeir and de Vrese, 2001). Fructo-oligosaccharides are prebiotic agents that are fermented by a number of colonic bacteria to modulate the growth of beneficial bacteria (Roberfroid, 2002). The number of *Bifidobacteria* has been shown to increase in the presence of inulin-type fructans with prebiotic properties. This increase occurs within a few days, but rapidly disappears upon withdrawal of the prebiotic compounds (after 1 week; Gibson and Roberfroid, 1995). The extent of increase in the number of *Bifidobacteria* is also dependent on their initial number in the gut. Breast-milk contains oligosaccharides with prebiotic properties that contribute to the increase in the number of *Bifidobacteria* after birth (Bode, 2009; Chichlowski et al., 2011).

Dietary fructans, which are present in various fruits and vegetables and added to food products, are used as an energy substrate by bacteria, including *Bifidobacterium* spp., that express β-fructofuranosidase, which promotes their development in the gut. A remarkable increase has been observed in the number of *Bifidobacterium* spp. in mice with diet-induced or genetically determined obesity that were supplemented with inulin-type fructans (Cani et al., 2007b). Interestingly, the number of *Bifidobacteria* was inversely correlated with the development of fat mass, glucose intolerance, and LPS level (Cani et al., 2007b). Inulin-type fructans increased the number of endocrine L cells in the jejunum and in the colon of rodents, and promoted the production and release of the active forms of GLP-1 and GLP-2 in the portal vein (Cani et al., 2004). GLP-1 participates in prebiotic-driven decreases in appetite, fat mass and hepatic insulin resistance, whereas GLP-2, as mentioned before, contributes to the reduced permeability of the intestinal wall and endotoxemia that are associated with obesity (Cani et al., 2006, 2009b). Interestingly, a 2-week treatment with inulin-type fructans (16 g per day) in healthy volunteers increased the postprandial release of gut peptides (namely GLP-1 and gastric inhibitory peptide; Cani et al., 2009a).

Cani and colleagues demonstrated that in rats fed a standard or high-fat diet, the addition of oligofructose to the diet reduced energy intake and consumption and protected against weight gain and fat-mass development, effects shown to be mediated by the modulation of endogenous gut peptides involved in appetite and weight regulation (Cani et al., 2004, 2005; Delzenne et al., 2005). The authors also reported that oligofructose increased the gut bifidobacterial content of high-fat diet-fed mice and that endotoxemia significantly and negatively correlated with *Bifidobacterium* species (Cani et al., 2007b). Parnell and Reimer (2009) randomized 48 otherwise healthy adults with a BMI > 25 kg/m^2^ to receive 21 g oligofructose or a placebo (maltodextrin) for 12 weeks. There was a reduction in body weight of 1.03 ± 0.43 kg with oligofructose supplementation, whereas the control group experienced an increase in body weight of 0.45 ± 0.31 kg over 12 weeks (*p* = 0.01). A lower area under the curve (AUC) for ghrelin (*p* = 0.004) and a higher AUC for peptide YY (PYY) with oligofructose (*p* = 0.03) coincided with a reduction in self-reported caloric intake (*p* > 0.05). Glucose decreased in the oligofructose group and increased in the control group between initial and final tests (*p* > 0.05).

### PROBIOTICS AND SYNBIOTICS

Probiotics have generated considerable interest in recent years because studies investigating their use in a variety of clinical conditions have yielded encouraging results (Floch and Montrose, 2005). Probiotics have been demonstrated to be beneficial in necrotizing enterocolitis, in adults and children with infective diarrhea and for the prevention and treatment of antibiotic associated diarrhea (Floch and Montrose, 2005; Hempel et al., 2012). Probiotics belonging to a number of genera including *Lactobacillus*, *Bifidobacterium*, *Saccharomyces*, *Streptococcus*, and *Enterococcus* (*Enterococcus faecium* SF68) have been used in these studies. The genus *Lactobacillus* comprises more than 90 species, the most commonly used include *L. acidophilus*, *L. rhamnosus*, *L. casei*, *L. bulgaricus*, *L. plantarum*, and *L. reuteri.* Most of the clinical trials reported to date have used blends of various probiotic genera, primarily *Lactobacillus* spp. in combination with other probiotics. The study of probiotics is complicated by the fact that the efficacy of these agents may be strain specific and the results from one probiotic (or combination) cannot be extrapolated to another. Furthermore, the results of clinical trials may depend on the potency (concentration) and the measures used to ensure the “bio-availability” of the bacteria. While probiotics are regarded as safe, few prebiotics have received the FDA GRAS (Generally Recognized as Safe) approval. Probiotics should be used with caution in critically ill and immunocompromised patients. In rare cases, probiotics have been associated with serious adverse effects in these patients including fungemia (*Saccharomyces boulardii*) and bacterial sepsis (Riquelme et al., 2003; Land et al., 2005). While clinical data supports the use of prebiotics and experimental data supports the use of probiotics, few studies have investigated the role of probiotics in patients with diabetes, insulin resistance, and obesity.

Luoto et al. (2010) randomized 159 women to receive *Lactobacillus rhamnosus* GG or placebo 4 weeks before expected delivery with the intervention extending for 6 months postnatally. Anthropometric measurements of the children were followed for 10 years. The perinatal probiotic intervention appeared to moderate the initial phase of excessive weight gain (up to 48 months), especially among children who later became overweight. Kadooka et al. (2010) conducted a multicenter, double-blind, randomized, placebo-controlled intervention trial in which subjects *(n* = 87) with an increased BMI (24.2–30.7 kg/m^2^) and abdominal visceral fat area (81.2–178.5 cm^2^) were randomly assigned to receive either fermented milk containing *Lactobacillus gasseri* SBT2055 (active FM; *n* = 43) or fermented milk without LG2055 (control FM; *n* = 44) for 12 weeks. Abdominal fat area was determined by computed tomography. In the active FM group, abdominal visceral and subcutaneous fat areas significantly (*p* > 0.01) decreased from baseline by an average of 4.6 and 3.3% respectively. Body weight and other measures also decreased significantly while, none of these parameters changed significantly in the control group.

Probiotics and synbiotics have been demonstrated to decrease intestinal permeability and endotoxemia in patients with liver disease and may serve as a model for reducing “metabolic endotoxemia” (Malaguarnera et al., 2010). In patients with minimal hepatic encephalopathy, Liu et al. (2004) demonstrated that treatment with a synbiotic significantly increased the fecal content of non-urease-producing *Lactobacillus* species at the expense of other bacterial species. Such modulation of the gut flora was associated with a significant reduction in blood ammonia levels, reversal of encephalopathy and a reduction in endotoxemia.

## CONCLUSION

Experimental and clinical data demonstrate that obesity is associated with changes in the intestinal microbiota. Furthermore, provocative data suggest that manipulation of the microbiome using prebiotics, probiotics, and synbiotics may reduce insulin resistance and fat accumulation. While probiotics are regarded as safe additional studies are required before such therapy can be widely recommended.

## Conflict of Interest Statement

The author declares that the research was conducted in the absence of any commercial or financial relationships that could be construed as a potential conflict of interest.
